# Effect of Nitrogen Partial Pressure on Structure, Mechanical Property, and Corrosion Behavior of ZrN_x_ Films Prepared by Reactive DC Magnetron Sputtering

**DOI:** 10.1155/2023/3604077

**Published:** 2023-04-10

**Authors:** Daoxuan Liang, Wei Dai

**Affiliations:** School of Electromechanical Engineering, Guangdong University of Technology, Guangzhou 510006, China

## Abstract

ZrN_x_ films were deposited by DC magnetron sputtering with pure Zr target in different nitrogen partial pressure atmospheres (*r* = N_2_/[Ar + N_2_]). The structure and composition of the thin films were characterized as a function of *r* using scanning electron microscope, glancing angle X-ray diffraction, and X-ray photoelectron spectroscopy. The hardness, adhesive strength, and corrosion behavior of the coatings were measured by nanoindentation, microscratch, and potentiodynamic measurements in 3.5 wt% NaCl solution. The results show that the structure of the ZrN_x_ films changes from a nearly stoichiometric ZrN with a typical columnar structure to mixed phases composited of ZrN and *α*-ZrN_x_ with a dense glass structure as *r* increases from 12% to 50%. The mechanical properties including hardness, elastic modulus, and adhesion decrease with increasing *r* due to nonstoichiometric compound and glass phase structure of the coatings, while the dense glass structure significantly improves the corrosion inhibition.

## 1. Introduction

Zirconium nitride (ZrN) based on transition metal nitrides has excellent mechanical and physical properties, such as high hardness, strong bonding, high melting point, excellent electrical and thermal conductivity, and remarkable biocompatibility [1]. Also, comparing to TiN, ZrN has higher hardness and elasticity modulus [2]. Nowadays, it has been widely used as a wear protection coating for cutting tools and mechanical components. ZrN is also available in a wide range of colors, so it has a wide range of prospects in the field of decorative coatings [3]. There are several ways to prepare ZrN coatings, such as vacuum cathodic arc evaporation plating [4, 5], DC reactive magnetron sputtering plating [6, 7], pulsed laser deposition [8], and ion beam assisted deposition [9].

By controlling the parameters of the coating deposition preparation process, such as the reaction gas pressure or the substrate bias pressure, different coating phase compositions can be obtained, which affects mechanical and chemical properties [10–12]. Meng et al. [8] studied the ZrN mechanical properties prepared by bias from -26.3 V to -400 V at 40% nitrogen partial pressure; Singh et al. [3] varied the deposition temperature to observe the effect of friction properties; Pilloud et al. [13] used RF magnetron sputtering method to control the bias voltage from 0 V to -160 V to study the morphological, mechanical, and optical property; Kuznetsova et al. [10] used an unbalanced magnetron sputtering system with controlled nitrogen flow at 0.5 Pa air pressure to study the crystal structure of zirconium nitride; Singh et al. [12] study the mechanical properties of ZrN prepared by different substrate temperatures. A series of ZrN_x_ films were prepared by Pei et al. [14] using reactive magnetron sputtering, varying [Ar]/([Ar] + [N_2_]). The effects of different nitrogen vacancy concentrations (*V*_N_ = 1–*x*, where *x* is the N/Zr ratio in ZrN_x_) on the mechanical properties and electrical properties of the coatings were compared. They found that the hardness increased from 18 ± 1.3 GPa to only 24 ± 1.2 GPa as *V*_N_ increased from 0 to a value of 0.24 and then decreased rapidly as *V*_N_ became greater than 0.30. Ruan et al. [15], using DC magnetron sputtering, compared ZrN_x_ coatings with increasing nitrogen from 0 to 5 sccm at 0.27 Pa, and they found that too high a background vacuum prevents the generation of ZrN_x_ in excess of the stoichiometric ratio.

It is clear that the structure and properties of the ZrN_x_ films deposited by PVD are sensitive to the deposition parameters (e.g., nitrogen partial pressure and bias). Accordingly, in this paper, the effect of nitrogen partial pressure on the structure, composition mechanical properties, and corrosion behavior of the ZrN_x_ films deposited by magnetron sputtering was studied with a wide range nitrogen partial pressure (from 12% to 50%). The relationships between of deposition parameter, microstructure, mechanical properties, and corrosion behavior of the ZrN_x_ coatings were discussed carefully.

## 2. Materials and Methods

The ZrN_x_ films in this experiment were prepared by DC magnetron sputtering coating system (Hua sheng MC800, China). A flat rectangular zirconium target were mounted on the magnetron target source (purity 99.4%), 500 mm in length and 100 mm in width. The samples are placed on a constant circumferential rotating table with motor rotating in 1 rpm. The distance between the target and the substrate is 80 mm when the substrate is rotated to be directly on the target surface. The substrate used for this experiment was cemented carbides (WC 6 wt.% Co) and silicon wafers (200). Before performing deposition, all substrates are placed in deionized water and cleaned with an ultrasonic cleaner for 30 minutes, and the remaining impurities on the substrate surface were remove. The substrate was then placed in an ethanol solution and cleaned by an ultrasonic cleaner for 30 minutes. The substrate is dried at the end of cleaning and transferred into the deposition chamber. The vacuum pump of the deposition chamber was turned on and pumped below 3 × 10^−3^ Pa. Argon gas (99.9% purity) is passed into the deposition chamber, and the bias value is set to -600 V for 20 minutes, with the aim of removing impurity gases adsorbed on the substrate surface. The next step is ion beam etching, where the bias voltage is set to -200 V in the deposition chamber as described previously, the ion source unit is turned on, and the current value is set to 10 A. The ion beam etching is performed for 20 minutes, which will further clean the substrate and increase the activation energy of the substrate surface. Then 250 sccm pure argon gas was introduced into the deposition chamber, and the air pressure was controlled at 0.5 Pa. The magnetron zirconium target was powered on, and the power was set to 4 kW to prepare a pure zirconium transition layer to improve the bonding of the coating. In the deposition step, the total chamber pressure is controlled to be 0.5 Pa. The nitrogen partial pressure *r* (*r* = N_2_/[Ar + N_2_]) was set between 12% and 50%. The ZrN_x_ film was produced by turning on the magnetron zirconium target power, setting the power at 4 kW, and depositing it for 150 minutes.

The scanning electron microscopy (SEM, Hitachi SU8220) was employed to obtain growth morphologies and thickness of the ZrN coatings. The grazing incidence X-ray diffraction (GIXRD, Bruker D8 Advance diffractometer) was carried out to determine the phase structure of as-deposited and oxidized films using a CuK*α* radiation source operated at 40 kV and 40 mA. The X-ray diffractograms were recorded with an incident angle of 1.0°, a scanning step of 0.02°, and a dwell time of 1.0 s. X-ray photoelectron spectroscopy (XPS, Thermofisher Escalab 250Xi) with a monochromatic AlK*α* source (hv = 148\6.6 eV) was adopted to analyze the chemical bonding states of the samples. The C1s peak at 284.8 eV was taken as a reference to calibrate the XPS spectra. Before commencing XPS analyses, the film surface was etched by an Ar^+^ beam with an energy of 3.0 keV and an irradiation area of 1.0 × 1.0 mm^2^ for 30 s to remove contaminations. Alk*α* (hv = 1486.6 eV) with 150 W power, and a 500 *μ*m beam spot was used. The binding energy is corrected with C1s = 284.8 eV. The spectrum is fitted using the Shirley function [16] to eliminate the background signal and the Gauss-Lorentz linearity to push convolution followed by split-peak fitting without data noise reduction smoothing, and the half-height width is controlled within 2.5 eV. Since there is orbital spin splitting in Zr [17], the Zr3d XPS consists of Zr 3d5/2 and Zr 3d3/2 with a binding energy difference Δ3d5/2 − 3d3/2 = −2.4 eV and an intensity area ratio Δ(3d5/2)/(3d3/2) = 3 : 2 [18]. The double peaks of the same component of Zr3d in Figure 1(a) due to spin splitting are labeled with the same color to avoid confusion.

The hardness and elastic modulus of ZrN films were measured by a nanoindentation tester (Anton Paar TTX-NHT^2^) with a Berkovich diamond indenter. In order to minimize the influence of the substrate on the hardness measurement, the penetration depth of the indenter was controlled below 10% of the film thickness to minimize the impact of the substrate. The loading and unloading rates were 20 mN/min, and the holding time at a peak load of 10 mN was 5.0 s. For each sample was tested repeatedly at 12 points. The adhesion strength of the films was tested via a nano scratch tester (Anton Paar RST) using Rockwell C diamond styli with a radius of 200 *μ*m. A normal load range of 1 N to 100 N, a scratch length of 3 mm, and a scratch speed of 3 mm/min were used in these experiments. Posttest characterization of the scratch-tested samples was performed using an optical microscope and a 3D optical surface profilometer.

The electrochemical corrosion behaviors of the bare and coated cemented carbides substrates (WC 6 wt.% Co) were investigated by open circuit potential (OCP) and potentiodynamic polarization test in an electrolyte cell, which consisted of a working electrode, a counter electrode (platinum sheet of 10 × 10 mm^2^) and a reference electrode (saturated calomel electrode, SCE). All the measurements were conducted on CHI660E electrochemical workstation in 3.5 wt% NaCl aqueous solution at room temperature. The coated and bare substrates were set as the working electrodes. The OCP measurement times of the bare and different coating substrates lasted for 400 s. The potentiodynamic polarization tests were carried out with a scan rate of 2 mV/min from -1.0 to +0.6 V versus OCP.

## 3. Results and Discussion

### 3.1. Morphology and Structure

Figure 2 shows the typical surface morphology and cross-section micrograph of the films deposited with *r* = 12% (Figures 2(a) and 2(b)), *r* = 30% (Figures 2(c) and 2(d)), and *r* = 50% (Figures 2(e) and 2(f)). It can be seen that the coating deposited with *r* = 12% shows a lattice surface topography and typical columnar cross-section (Figures 2(a) and 2(b)). The film is consisted of two layers: a ZrN_x_ layer with a thickness of about 831 nm and a Zr interlayer with a thickness of about 300 nm. The growth structure of the ZrN_x_ films refines gradually with increasing the nitrogen partial pressure. The ZrN_x_ film deposited at the nitrogen partial pressure of 50% shows a typical glass phase structure without any feature (Figure 2(f)). In the meantime, the thickness of the ZrN_x_ layer showed a significant decrease from 831 nm to 343 nm with the increase of the partial pressure of nitrogen. On the one hand, the increase the increase of the reaction gas N_2_ causes the target poison and thus decreases the deposition rate [12]. On the other hand, for metal target, Ar has higher sputtering yield compared to N_2_. Therefore, the decrease of Ar partial pressure would decrease the growth rate of the ZrN_x_ layer.

The GIXRD test results of ZrN_x_ are presented in Figure 3 for a typical NaCl structure. The ZrN (PDF #71-4633) prepared at *r* = 12 ~ 50% all shows (111), (200), (220), and (311) orientations, in which (111) and (200) peaks are more obvious. References indicated that (111) and (200) are the main weaving of the cubic phase of ZrN [10], indicating that all ZrN coatings have significant crystallization. The ZrN_x_ prepared at 12% to 50% partial pressure of nitrogen are mainly (200) crystalline orientation. With the increase of nitrogen partial pressure, the peak shape broadens, and the peak intensity decays. In particular, as the partial pressure of nitrogen increases, the (200) selectively oriented peak shows a clear downward trend, and the (110) peak disappears. It has been shown that the microcrystal size of ZrN_x_ decreases with increasing nitrogen partial pressure because the structure grows toward disorder and tends to amorphization [12]. Comparing the ZrN standard cards, it can be found that as the partial pressure of nitrogen increases, the coating preference peak shifts to a high angle, indicating a shift from compressive stress (*r* ≤ 30%) to tensile stress (*r* > 30%) in the coating, and various studies support this change phenomenon [19, 20]. This peak-shifting phenomenon will also lead to a decrease in the hardness of the coating, which will be discussed in Section 3.2. Some weak peaks ascribed to pure zirconium are also detected in the XRD pattern. The presence of Zr peaks mainly originates from the pure metal Zr interlayer.

The typical chemical states of the films are analyzed with using XPS. The chemical valence states of Zr3d and N1s for *r* = 12%, 30%, 50% are shown in Figures 1(a) and 1(b), respectively. The presence of O is observed in all films prepared at partial pressure after etching in the Zr3d patterns (ZrO_2_) because the Ar^+^ gas used for etching, even though it is chemically inert, changes the original concentration distribution in the sample when used for etching, as the high-energy Ar^+^ bombardment reorients the film atoms [21, 22]. The O content detected ranged from 9.6 at% to 9.2 at%. And it has been pointed out that N atoms are preferentially sputtered relative to O atoms, so the residual N/O concentration ratio of the sample after sputtering will be larger than that of the initial sample. Three main products are presented in the Zr3d spectrum, component #1-ZrN: 179.2 to 180.3 eV; component #2 *α*-ZrN_x_ (amorphous ZrN_x_): 180.3 to 180.7 eV; and component #3-ZrO_2_: 182.2 to 182.4 eV [8, 10, 23–25]. It can be observed that as the partial pressure of nitrogen increases, the initial peak of Zr3d moves from low to high binding energy, and component #2 appears and gradually increases, the content of component #1 gradually decreases, and the relative content of Zr^4+^ oxides corresponding to component #3 remains unchanged.

At room temperature, according to the law of thermodynamics, the ZrO_2_ phase is preferred over the formation of ZrN metallic zirconium (Δ*H*_*f* *ZrO*2_° : −1042.8 kJ/mol, Δ*H*_*f* *ZrN*_° : −365.5 kJ/mol). There has been controversy about the determination of component #2. Del Re et al. [26] deposited the ZrN films by reactive magnetron sputtering with different nitrogen partial pressures and found that three products were observed in the N1s narrow sweep spectrum at (a) 397.1 eV, (b) 396.4 eV, and (c) 395.8 eV, where product (b) corresponds to the product of the N1s peak in this paper. The products (b) and (c) reported in the paper correspond to the state of ZrN over stoichiometric ratio, where it is determined that product (c) is ZrN_2_. While the authors argue that the N/Zr of the as-deposited ZrN film is below 1, denying the presence of Zr_3_N_4_. However, Rizzo et al. [27] prepared the ZrN_x_ films by RF magnetron sputtering, and they observed the simultaneous presence of ZrN_2_, Zr_3_N_4_, and ZrN at 100% nitrogen partial pressure, and their binding energies were located at 395.4 eV, 396.5 eV, and 397.3 eV in the N1s pattern, respectively. Carvalho et al. [28] prepared the ZrN_x_ films by reactive magnetron sputtering and also believed that the product under this binding energy peak position is Zr_3_N_4_. Therefore, in this paper, combining the stoichiometric ratio and binding energy, it can be judged that the component #2 might be an amorphous ZrN_x_ (*α*-ZrN_x_) which belongs to the substable state with an overstoichiometric ratio (such as ZrN_2_ and Zr_3_N_4_) [26, 29]. It can be seen that the *α*-ZrN_x_ cannot observed in the low nitrogen partial pressure environment. As the partial pressure of nitrogen increased, GIXRD indicates that the film became amorphous, and the XPS shows that the component #2 (*α*-ZrN_x_) increases while component #1 (ZrN) decreases, implying the appearance of substable products in the films.

In the plot of N1s, component #1 ZrN compound lies in the range of 397.2~397.7 eV [27], while component #2 is in the interval of 395.8~396.1 eV. It can be observed that from *r* = 12 to *r* = 30, the N1s peak is significantly distorted, and the new product can be obtained by deconvolution, which is in accordance with the phenomenon observed for Zr3d, and the component #2 increases significantly with the increase of the nitrogen partial pressure.

### 3.2. Mechanical Properties

The hardness and elastic modulus of the ZrN coatings are shown in Figure 4. The hardness and elastic modulus of the ZrN_x_ film (*r* = 12%) at stoichiometric ratio are about 23 GPa and 391 GPa, respectively. The hardness and elastic modulus reach the maximum values of 26.5 GPa and 379.5 GPa at *r* = 20%, respectively, and then decrease to about 14 GPa and 283 GPa with increasing nitrogen partial pressure. The SEM images (Figure 2) show that the grain size of the as-deposited ZrN_x_ films gradually decreases with increasing partial pressure of nitrogen. Grain refinement could enhance the mechanical properties of the films [30]. However, the XRD and XPS analyses indicate that the films change from columnar crystalline to the amorphous structure as well as from isometric to overmetric ratios, causing the reduction of the hardness. The two conflicting factors cause the film hardness and elastic modulus to increase firstly and then decrease with the partial pressure of nitrogen.

The optical morphology of the scratches of the ZrN_x_ films prepared with different partial pressures of nitrogen is shown in Figure 5. In this experiment, the load values corresponding to the three main failure events are marked as critical loads (Lc) [31], where Lc_1_ corresponds to the initial scratch in the scratch track, Lc_2_ corresponds to the first appearance of a defect within the scratch track and can measure the cohesive bond strength of the coating [32], and Lc_3_ corresponds to the complete loss of the coating and exposure of the substrate. As the partial pressure of nitrogen increases, the adhesion of the films tends to decrease gradually, and the result is close to the trends of the hardness and elastic modulus. At *r* = 12%, its Lc_3_ value is 36 N and the Lc_3_ value drops to 23 N at *r* = 50%. Within the scratch tracks of all results, only small tensile cracks appear before the coating flakes off, there is no crack growth or stacking, and there is no brittle flaking at the edges of the scratch tracks, i.e., the films have good adhesion. The difference in the scratch performance of the ZrN_x_ films might be attributed to the film hardness and elastic modulus.

### 3.3. Corrosion Behavior

Figure 6(a) presents the evolution of the OCP curves of the bare cemented carbides and coated samples in a 3.5 wt% NaCl solution for 400 s. The average potential of the bare substrate sample was -0.374 V. Variations in the OCP curves of the coated samples show a similar trend, except for the film deposited with *r* = 12%, which has a strong initial fluctuation. The corrosion potential of the film material corresponded to the initial high potential in the OCP curves.  Figure 6(b) shows the potentiodynamic polarization curves of different nitrogen partial pressure of ZrN_x_-coated and bare substrates in a 3.5 wt% NaCl aqueous solution at room temperature. As shown in Figure 6(b), the corrosion resistance of the bare cemented carbides substrate has been significantly improved by applying the films, especially for the *r* = 40% ZrN_x_-coated sample. The bare cemented carbides substrate exhibits the most negative *E*_corr_ (-0.64 vs. SCE) and highest *I*_corr_ (8.44 *μ*A/cm^2^) among the samples. After being coated with ZrN_x_, the sample shows a great improvement of corrosion resistance that the *I*_corr_ (0.2~0.7 *μ*A/cm^2^) is one order magnitudes lower than the bare sample. The desirable performance was attributed to the dense ZrN_x_ coating, which increased energy barrier for corrosion media [33]. However, changing the nitrogen partial pressure of coatings shows a great difference in corrosion resistance. The parameters of *I*_corr_ differ by a factor of two or three and fluctuate with the increasing of the nitrogen partial pressure.

## 4. Conclusions

In this paper, the ZrN_x_ films were deposited by DC magnetron sputtering. The influence of the nitrogen partial pressure on the structure, composition, mechanical properties, and corrosion behavior of the ZrN_x_ films was researched. It is found that the nitrogen partial pressure has significant effect on the microstructure and chemical composition of the ZrN_x_ films. As the nitrogen partial pressure increases, the structure of the ZrN_x_ coatings changes from a nearly stoichiometric ZrN with typical columnar structure to mixed phases composited of crystal ZrN and *α*-ZrN_x_ with a dense glass structure. The stoichiometric ZrN_x_ film deposited with the nitrogen partial pressure of 20% shows the maximum values of hardness and elastic modulus. At other nitrogen partial pressures, the nonstoichiometric compound and glass phase structure cause the decrease of the hardness and elastic modulus. However, the dense glass structure can significantly improve the corrosion inhibition of the ZrN_x_ films.

## Figures and Tables

**Figure 1:** High-resolution XPS spectrum of (a) Zr3d and (b) N1s of the films prepared at different partial pressures of nitrogen.

**Figure 2:** (a, c, e) Typical surface morphology and (b, d, f) cross-section morphology of the ZrN_x_ films deposited with (a, b) *r* = 12%, (c, d) *r* = 30%, and (e, f) *r* = 50%.

**Figure 3:** GIXRD patterns of the ZrN_x_ films prepared at different partial pressures of nitrogen.

**Figure 4:** Hardness and elastic modulus of the coatings prepared at different partial pressures of nitrogen.

**Figure 5:** The adhesion of the coatings prepared at different partial pressures of nitrogen.

**Figure 6:** (a) The open circuit potential and (b) potentiodynamic polarization curves of bare and coated samples.

## Data Availability

The data used to support the findings are available from the corresponding author upon request.
